RETRACTED

# The evolution of renewable energy environments utilizing artificial intelligence to enhance energy efficiency and finance

**DOI:** 10.1016/j.heliyon.2023.e16160

**Published:** 2023-05-11

**Authors:** Fengge Yao, Zenan Qin, Xiaomei Wang, Mengyao Chen, Adeeb Noor, Shubham Sharma, Jagpreet Singh, Dražan Kozak, Anica Hunjet

**Affiliations:** a Finance of School, Harbin University of Commerce, Harbin, China; b School of Tourism and Culinary Arts, Harbin University of Commerce, Harbin, China; c School of Media, NingboTech University, Ningbo, 315000, China; d Department of Information Technology, King Abdulaziz University, Jeddah, 80221, Saudi Arabia; e Mechanical Engineering Department, University Centre for Research and Development, Chandigarh University, Mohali, Punjab, 140413, India; f School of Mechanical and Automotive Engineering, Qingdao University of Technology, 266520, Qingdao, China; g Department of Computer Science and Engineering, IK Gujral Punjab Technical University, SAS Nagar, Punjab, 160055, India; h University of Slavonski Brod, Mechanical Engineering Faculty in Slavonski Brod, Trg Ivane Brlić-Mažuranić 2, HR-35000, Slavonski Brod, Croatia; i University Center Varaždin, University North 104. Brigade 3, HR-42 000, Varaždin, Croatia

**Keywords:** Artificial intelligence, Energy efficiency financing, Renewable energy, G7 economies

## Abstract

The development of a country is inseparable from the material guarantee mainly based on energy, but energy is limited, which may restrict the sustainable development of the country. It is very necessary to accelerate the adoption of programs aimed at switching non-renewable energy sources to ones that are, and giving priority to improving renewable energy consumption and storage capabilities. From the experience of the G7 economies, the development of renewable energy (RE) is inevitable and urgent. The China Banking Regulatory Commission has recently issued a number of directives, such as the “Directives for Green Credit” and “Instructions for Granting Credit to Support Energy Conservation and Emission Reduction,” to help businesses that use “renewable energy expand”. This article firstly discussed the definition of the “green institutional environment” (GIE) and the construction of the index system. Then, on the basis of clarifying the relationship between the GIE, and RE investment theory, a semi-parametric regression model was constructed to empirically analyze the mode and effect of the GIE. Considering the balance between improving model accuracy and reducing computational complexity, the number of hidden nodes opted in this study is 300 so as to lower the time needed to predict the model. Finally, from the perspective of enterprise scale, the level of GIE played a significant role in promoting RE investment in small and medium-sized enterprises, with a coefficient of 1.8276, while the impact on RE investment in large enterprises had not passed the significance test. Based on the conclusions, the government should focus on building a GIE dominated by green regulatory systems, supplemented by green disclosure and supervision systems, and green accounting systems, and should make reasonable plans for releasing various policy directives. At the same time, while offering full play to the guiding role of the policy, its rationality should also be paid attention to, and the excessive implementation of the policy should be avoided, so that an orderly, and good GIE can be created.

RETRACTED

## 1 Introduction

### 1.1 Background meaning

Under the background of sustainable development, the green economy has gradually become the main development direction of various countries, and its essence lies in achieving sustainable economic development with coordinated development and environmental friendliness as the core. In order to achieve sustainable development, it is now imperative to invest in renewable energy. However, in practice, commercialization and industrialization have nourished people's egotistical desires, methods of dominance and control, and stymied the development of renewable energy, undermining the equilibrium between humanity and nature as well as between individuals. At the same time, the economic uncertainty of the value of resources and the environment and the unpredictability it brings make sustainable development encounter a very difficult theoretical problem. As a comprehensive evaluation of environmental economic policies, GIE has both “green” and “policy” attributes, and the resulting environmental and economic benefits can affect RE investment. However, as the current GIE system is composed of many elements, studying the impact of the GIE system and various environmental and economic policies on RE investment is of great help to clarify the key elements and effects of GIE and objectively locate the focus and direction of policies. In this way, a systematic GIE system can be formulated, effectively deal with the derived problems in the development of RE, and comprehensively promote the transformation and development of energy strategies. This paper adopts the method of group estimation for the impact of enterprises of different sizes and different industries on renewable energy, and elucidates some of the implications of renewable energy on enterprises and various industries. The study is prospective, but the experimental results still lack a certain representativeness. On the basis of clarifying the relationship between GIE and RE investment theory, a semi-parametric regression model is constructed, and the model and effect of GIE are analyzed empirically.

RETRACTED

On the basis of clarifying the relationship between GIE and renewable energy investment theory, this paper innovatively builds a semi-parametric regression model to empirically analyze the model and effect of GIE. This paper further estimates the effect of GIE and various green economic policies on RE investment based on the industry and enterprise scale. The differences and effectiveness of the GIE for RE companies of different scales and industries are clarified, and it can provide some valuable advice for future related research. While giving full play to the guiding role of the policy, this paper should also pay attention to its rationality and avoid excessive implementation of the policy, so as to form an orderly and good GIE.

## 2 Related work

RE is a kind of clean energy. Samadi P [1]. used approximate dynamic programming to create running schedules for different types of devices, either mandatory or supervised. Rezaei R [2]. studied decision-making models for the use of RE in agriculture in Iran. The inclusive principle of technology adoption and use was the researcher's main focus. They expanded it to look at the factors that affect the decision to use RE. A hybrid cascade topology with three phases was proposed by RR Karasani [3] and reduced costs, losses, installation space, voltage, and the circuit breaker's inverter. A decentralized system for a group of intelligent homes is referred to as a smart community. Yang L [4] used smart home planning technology that allowed customers to automatically plan energy loads for different uses, and modern home planning was often implemented in a decentralized manner within smart communities, as consumers competed for RE at the community level due to low costs. These scholars have researched on RE, but there was no actual research process.

Artificial intelligence is an important aspect of computer science. Among them, A deeper understanding of physical theory, in the opinion of Hassabis D [5], can significantly aid in the creation of intelligent devices. He looked at the relationship between artificial intelligence and neuroscience over time and focused on the most recent developments in AI that have influenced research on human and other animal neuro-computing. 5G mobile networks were considered to be a key factor in the ICT industry and offered different services and met different needs. Rongpeng [6] attempted to demonstrate an important aspect of the technological revolution in the 5G era, including radio infrastructure, navigation systems, service delivery systems, etc. The impact of the industrial and digital revolutions has had a huge impact on almost everything. Makridakis S [7] discussed the achievements of the industrial, digital and information revolutions, and believed that this goal could bring about major changes affecting all aspects of the world and life. Modern malware used high-tech methods to hide passive and active scanning tools. Therefore, Caviglione L [8] aimed to detect cryptomal ware using two smart tool-based detection methods. These scholars have used artificial intelligence algorithms to conduct research, but they did not specifically target a certain aspect and lack pertinence.

RETRACTED

## 3 RE prediction model based on artificial intelligence

### 3.1 Status quo of RE development

#### 3.1.1 Wind energy

According to the theorem obtained from physical research, the energy of the wind generated by the air flow on the earth, when it passes through a certain section in a very short period of time, can be obtained according to this formula:

(1) $$F=\frac{1}{2}nv^{2}=\frac{1}{2}\alpha Erv^{3}$$

The renewable energy (RE) model starts with book value and takes into account premium as the rise in asset value, which is represented by residual income. The model that measures the increase in value according to residual income is called the residual income model. It can be applied to the valuation of common shares. In formula (1), α represents the air density; E represents the area of the section taken when calculating wind energy; r represents the time span of the observer to measure the wind energy, and v represents the instantaneous wind speed in this very short period of time [9].

The wind-turbine hits its blades through air molecules, captures wind energy and converts it into the potential energy of the rotation of the wind-turbine blades. The final input power to the wind-turbine can be calculated by this formula:

(2) $$Q_{w}=0.5\alpha \pi T^{2}D_{q}\left(\eta ,\gamma \right)v^{3}$$

Informula (2), $D_{q}$ represents the conversion coefficient of wind energy, which is affected by the actual values of η and γ of different fans. Under ideal conditions, the maximum value can reach 0.593, that is, the conversion rate of wind energy can reach 59.3% under ideal conditions. However, in the actual “wind-power generation system”, due to the combined action of various constraints and influencing factors, the actual $D_{q}$ value is often less than 0.5, that is, the actual conversion efficiency is less than 50%. Fig. 1 shows a diagrammatic representation of the production of wind energy.

**Fig. 1:** Illustration of wind power generation.

RETRACTED

Due to the complex external environmental factors, many input variables and large scale of model parameters in wind speed prediction, the traditional neural network model cannot achieve the purpose of accurate prediction [10].

#### 3.1.2 Solar energy

Due to the absorption of a large amount of photon energy, the electrons on the Q junction side and the holes on the N junction side are excited and move toward each other, resulting in a potential across the QN junction. In the ideal state, the solar cell can be approximately equivalent to a constant current power supply $L_{qh}$, a diode C in parallel, a leakage resistance $T_{oh}$ in parallel, and a material resistance $T_{o}$ in series. According to Kirchhoff's law, the calculation formula for the load characteristics under ideal conditions can be obtained as:

(3) $$L=L_{qh}-L_{C}-L_{oh}$$

(4) $$L_{C}=L_{0}\left(e^{\frac{p\left(U+LT_{o}\right)}{kR}}-1\right)$$

(5) $$L_{oh}=\frac{U+T_{o}L}{T_{oh}}$$

In formulas (3) (4) (5), L and T represent the output current and voltage of the photovoltaic cell, respectively, and k is the thermodynamic Boltzmann constant.

#### 3.1.3 Tidal energy

At present, a relatively mature technology to extract tidal energy from the movement of ocean currents is to build reservoirs on the coast and use the water level difference between the two sides of the reservoir during daily high and low tides to guide seawater to impact the generator in the dam of the reservoir and drive the generator blades to rotate to generate electricity [11].

In the ideal state, according to the physical mass conservation formula and Euler's theorem, the formula of the normal phase driving force generated by the seawater flow on the turbine blades is:

(6) $$E=n\left(U_{1}-U_{2}\right)$$

In formula (6), n is the mass of seawater, and $U_{1}$ and $U_{2}$ are the water flow velocity at the far end of the turbine inlet side and the far water flow velocity at the turbine outlet side, respectively.

At this time, using the physics Bernoulli formula, the pressure drop ΔQ on both sides of the turbine can be obtained as follows:

(7) $$\Delta Q=\frac{1}{2}\alpha \left(U_{1}^{2}-U_{2}^{2}\right)$$

Then the thrust E received by the turbine in area B is:

(8) $$E=\Delta QB=\frac{1}{2}B\alpha \left(U_{1}^{2}-U_{2}^{2}\right)$$

The kinetic energy F when the seawater with a certain length i is controlled to flow through the turbine can be expressed as:

(9) $$F=\frac{1}{2}nU^{2}=\frac{1}{2}\alpha BiU^{2}$$

Then the corresponding power Q is:

(10) $$Q=\frac{F}{r}=\frac{1}{2}\alpha B\frac{1}{r}U^{2}=\frac{1}{2}\alpha BiU^{3}$$

### 3.2 Common prediction models

At present, the most common forecasting scheme with a wide range of applications is the forecasting based on time series, including traditional physical and mathematical models, artificial intelligence models and hybrid models [12].

RETRACTED

#### 3.2.1 Moving average model

The moving average model $x_{r}$ is expressed as:

(11) $$x_{r}=\alpha_{0}+\mu_{1}x_{r-1}+\mu_{2}x_{r-2}+...+\mu_{q}x_{q-2}+\eta_{r}-\alpha_{1}\eta_{r-1}-\alpha_{2}\eta_{r-2}-...-\alpha_{p}\eta_{r-p}$$

#### 3.2.2 Neural network model

The neural network model is inspired by the brain systems of biological entities, that is, by the cooperation of many interconnected neurons to solve various problems, including the process of human learning problems. A Neural network is a mathematical prediction model that can undertake perform different functions. It can configure the parameters of the model network based on different types of tasks, including continuous data prediction, to complete different prediction tasks [13]. The main model parameters of the neural network model are the “connection-weight”, and “offset of the hidden-nodes in the hidden-layer”, “the activation-function of the hidden-layer”, and “the connection-weight”, and “offset of the output-layer”.

The mathematical expression of a single-layer neural network model can usually be written as:

(12) X=αf(W⋅Y+A)+a

In formula (12), Y and X are the “input-layer”, and “output-layer data” of the “neural network model”, respectively.

#### 3.2.3 Support vector machine-model

The “support-vector machine” is transformed into a dual optimization problem by introducing Lagrangian coefficients into the hyperplane mathematical model, which is expressed as:

(13) $$\overset{\min}{w,a},\overset{\max}{b}H\left(w,a,b\right)=\frac{1}{2}{\left\|w\right\|}^{2}-\sum_{j=1}^{m}\beta_{j}\left[x_{j}\left(w\cdot y_{j}+a\right)-1\right]$$

H(w,a,b) is the Lagrangian function and $\beta_{j}$ is the Lagrangian coefficient.

After solving the dual optimization problem, the mathematical formula of its optimal decision-making process, that is, the final prediction model with the smallest prediction error, is as follows:

(14) $$h\left(y\right)sgn\left(f\left(y\right)\right)=sgn\left(w_{0}\cdot y+a_{0}\right)=sgn\left(\sum_{j=1}^{m}\beta_{j}^{*}x_{j}\left(y_{j}y\right)+a_{0}\right)$$

### 3.3 Extreme learning machine (ELM) model

#### 3.3.1 ELM algorithm principle

Since the connection weights and hidden layer offsets are randomly selected, the forward artificial neural network can be simplified into a linear system. Only by performing the matrix generalized inverse operation on the input-layer and output-layer data, the output layer weights of the forward artificial neural network can be determined to determine the network parameters of the entire model. Fig. 2 shows the network structure of the ELM.

RETRACTED

**Fig. 2:** ELM network structure.

This learning algorithm greatly reduces the amount of computation required to train the model while ensuring the approximation accuracy, effectively reduces the time required to determine network parameters, and overcomes the shortcomings of traditional learning algorithms [14].

For a given training set $D_{train}$ consisting of M training samples ${\left\{\left(y_{j},r_{j}\right)\right\}}_{j=1}^{M}$, the ELM mathematical model can be obtained:

(15) $$\sum_{j=1}^{\tilde{M}}\beta_{j}f_{j}\left(y_{j}\right)=\sum_{j=1}^{\tilde{M}}\beta_{j}f\left(w_{j}y_{j}+a_{j}\right)={\tilde{r}}_{j}$$

(16) $$\sum_{j=1}^{M}\left\|{\tilde{r}}_{j}-r_{j}\right\|=0$$

$\tilde{M}$ is the “number of hidden-nodes in the hidden-layer” of the “predictive model”; f(x) is the “activation function of the hidden-layer” of the “predictive model”, and $a_{j}$ is the “offset from the input-layer to the jth hidden-node of the hidden-layer”.

$$\sum_{j=1}^{\tilde{M}}\beta_{j}f\left(w_{j}y_{j}+a_{j}\right)=r_{j}$$

Gβ=R

$$G=\left[\begin{array}{l} f\left(w_{1}y_{1}+a_{1}\right)...f\left(w_{\tilde{M}}y_{1}+a_{1}\right)\\ ...\\ f\left(w_{1}y_{M}+a_{1}\right)...f\left(w_{\tilde{M}}y_{M}+a_{\tilde{M}}\right) \end{array}\right]$$

$$\beta =\left[\begin{array}{l} \beta_{1}^{R}\\ .\\ .\\ .\\ \beta_{\tilde{M}}^{R} \end{array}\right]$$

$$R=\left[\begin{array}{l} r_{1}^{R}\\ .\\ .\\ .\\ r_{M}^{R} \end{array}\right]$$

#### 3.3.2 Adjustment of structural factors of the ELM model

First, considering the variables of the ELM model, according to the characteristics of the target analyzed in this study, the activation function and network structure of the model are modified to enhance the model's accuracy. Since the samples in the test set are not visible before prediction, ELM first trains the model parameters in the training set, and then evaluates the prediction performance of this parameter set based on the performance of the validation set.

##### 3.3.2.1 The influence of the ELM activation function on the prediction results

In the research process, MATLAB software is mainly used to simulate and compare the prediction models under different activation functions. Compared with the “root mean square error (RMSE)”, the results are shown in Fig. 3.

**Fig. 3:** RMSE error of ELM prediction model under different activation functions.

By comparing the different curves of the outcomes illustrated in Fig. 3, it can be observed that the use of different activation functions has a greater impact on the error of the prediction model output. Among them, the sigmoid function of sigmoid has the best performance and is suitable for prediction cases, and has obvious advantages over the other two functions in terms of activation.

RETRACTED

##### 3.3.2.2 The implications of the number of hidden-nodes in ELM on the prediction results

Evaluating the appropriate number of hidden-nodes and selecting an appropriate activation function are crucial when configuring the network structure factors of the ELM learning machine. The use of the sigmoid function was determined based on the research content of Fig. 3. By changing the number of hidden-nodes in the MATLAB simulation software, the prediction findings of the training-set and the validation-set are obtained, and the RMSE with the actual value is used to calculate the error. The model performance with the different numbers of hidden nodes is shown in Fig. 4.

**Fig. 4:** RMSE error of ELM prediction model with the different number of hidden-nodes.

Fig. 4 exhibits that the RMSE of the training-set and test set depends on the number of different hidden nodes, and it could be seen that as the number of hidden-nodes rises, the training-set also increases. The RMSE on the training-set reduces first and then slowly, while the RMSE on the validation set decreases rapidly when the number of hidden-nodes is less than 200. When the number of hidden-nodes is between 200 and 500, it remains stable. When the number of hidden-nodes is more than 500, there is a clear increasing trend. Considering the balance between improving model accuracy and reducing computational complexity, the number of hidden-nodes selected in this study is 300 so as to lower the time needed to predict the model.

## 4 Energy efficiency financing and RE development in G7 economies

### 4.1 RE under the green regime

#### 4.1.1 Investment in RE

For the concept of RE investment, it is mainly defined from macro and micro perspectives. From a macro perspective, RE investment is: social capital flowing to the field of RE, including investment in new projects and expansion of existing projects. However, investment in the research and development sector and investment in manufacturing are not included [15]. From a micro level, most of them take enterprises as the main body to define RE investment. These definitions distinguish the main body, object, purpose, and result of the investment.

#### 4.1.2 GIE

Under the background of sustainable development, the government has implemented a series of policy measures. It is worth noting that these policy instruments all have a common feature, that is, the “green” attribute. In fact, the government has virtually constructed an institutional environment with “green” attributes, and the construction of this institutional environment can inevitably have an impact on economic life [16]. GIE refers to various policy means and institutional arrangements that can promote green development to encounter the demands of evolution of sustainable growth.

RETRACTED

#### 4.1.3 The mechanism of the GIE on RE investment

Fig. 5 shows the mechanism of the GIE on RE investment.

**Fig. 5:** The mechanism of GIE on RE investment.

### 4.2 Construction of GIE index

#### 4.2.1 GIE system

The Green policy has the function of guiding the country's green development and institutional guarantee. The GIE consists of three modules: “ex-ante control”, “in-process governance”, and “ex-post accounting”. From a hierarchical point of view, the main considerations are as follows. Endogenous growth theory challenges the assumption of exogenous technology in neoclassical growth theory, holds that technological progress is an endogenous variable, and thus explains the rationale causes for variations in economic growth rates are examined, and the prospect of future economic growth is investigated. Endogenous growth theory also holds that endogenous variables are sensitive to and affected by policies (especially fiscal policies). Economic entities, especially the fiscal policies made by the government, will affect economic growth.

1) Under the green supervision and disclosure system, there are three secondary indicators, including the green label system and the green market access system. The green label system refers to the inspection of green enterprises and green products produced through a series of procedures, and those that meet the standard conditions receive corresponding labels; the green market access system refers to establishing some special markets and artificially controlling some “green” enterprises or products that do not meet the regulations from the market by setting certain standards and conditions. The term environmental information disclosure system refers to the policy system that enterprises need to clearly disclose corporate accounting information to the outside world according to the unified regulations of the country [17].
2) There are five secondary indicators under the green norm system, including the performance appraisal system and the environmental management system. The performance appraisal system has increased the importance of environmental indicators and played an important role in environmental responsibility [18]. Green economic policies are a set of government policies based on the traditional industrial economy, aiming to achieve harmonious development of the economy and the environment.
3) There are four secondary indicators under the green accounting system, including green GDP and emission trading market. “Green auditing” refers to monitoring a company's policies and systems related to environmental norms. “Green accounting” is a system that incorporates environmental information into accounting subjects related to environmental protection for reasonable statistics and reporting. Green GDP aims to incorporate environmental and resource factors into the GDP measurement system, thus achieving a critical evaluation of ecological and economic merits. The development of artificial intelligence (AI) technology has obtained a broad space, the introduction of AI in the domain of econometric research, as well as the improvement of machine learning algorithms can have a substantial implication on econometrics. Modern economic theory fails to explain the emergence, development, and evolution of economic systems, but the usage of AI technology can effectively improve the economic theory in the interpretation of the real economy, and provide reliable economic and social policies.

RETRACTED

#### 4.2.2 Measurement of GIE index

##### 4.2.2.1 Index system

Combined with the current development of GIE work, and based on the four factors considered in the selection of indicators, relevant indicator data were selected [19].

##### 4.2.2.2 Index level measurement

###### 4.2.2.2.1 Dynamic weight analysis of indicators

To obtain the GIE index, it is necessary to combine the weight curve and the index curve of each index. It is generally a combination of subjective and objective empowerment methods. This is taking into account the data characteristics of the indicators, and at the same time, there are subjective judgments for individual indicators; it does not completely rely on data, which is not entirely subjective judgments.

###### 4.2.2.2.2 Indices level measurement

By synthesizing the size and weight of each index, the changes in the GIE index from 2008 to 2016 are obtained, as shown in Fig. 6.

**Fig. 6:** Changes in the GIE index.

It can be seen from Fig. 6 that on the whole, the GIE index is on the rise, with a range of [0.2–0.8]. However, the GIE index suddenly showed a downward trend in 2011 [20]. From a time, point of view, there were many major events in 2010–2011, and these events caused the government's policy focus to shift to a certain extent; in addition, in 2016, the GIE index rose faster.

### 4.3 Examination of the role of GIE in affecting RE investment

#### 4.3.1 Variable selection and description

##### 4.3.1.1 Selection of variables and data sources

In addition to the impact of the GIE on RE investment, the factors that affect RE investment should also be considered from the perspective of enterprises themselves. Based on the previous analysis, several variables are selected here as shown in Table 1.

RETRACTED

**Table 1:** A portrayal of the primarily factors and indicators.

	Variable	Symbol	Indicator description
1	Investment in RE	INV(Investment)	The sum total of cash that renewable energy (RE) companies have paid out for the procure/purchase and advancement of tangible, intangible, and other long-term value assets.
2	GIE level	INDEX	GIE Index
3	Enterprise resource endowment	RE (Re-lending)	Asset-liability ratio of RE companies
4	Business age	AGE	List of RE companies
5	Development potential	TQ (Tobin's)	Tobin-Q value of RE companies

For variables, given the availability of data, the GIE index is a macro index, while the data of other variables belongs to each sample enterprise.

##### 4.3.1.2 Mathematical/numeric statistics analysis of variables

Table 2 is a description of each variable.

**Table 2:** Statistical description of each variable in 2008–2018.

variable	average	median	minimum	maximum value	standard deviation	skewness	kurtosis
INV	951900000	232300000	−35200000	27960000000	2449148000	6.7107	54.8628
INDEX	0.5169	0.5540	0.1305	0.8547	0.2171	−0.1993	−1.2458
RE	0.5571	0.5712	0.0386	1.2008	0.1788	−0.3268	0.0490
AGE	13.47	14.00	0.00	28.00	5.4130	−0.0199	−0.4987
TQ	1.7340	1.4590	0.7978	10.1589	0.9337	3.1969	16.2706

Table 2 reflects that,

①. In the sample-interval, from the “maximal value”, “minimal value”, and “standard deviation” of RE investment, it can be seen that the degree of dispersion of RE investment data is high. Further, the skewness value of RE investment is 6.7107, and the kurtosis value is 27.7687, indicating that the sample-data presents a “right-skewed distribution”, and the distribution shape presents a sharp peak.

②. The mean and median of the environmental level of green institutions are relatively close, and it can be observed from the “standard deviation” that the sample data has little difference, the value range is small, and the data is relatively concentrated. Further, the skewness value of the GIE level is −0.1993, and the negative sign indicates that the overall sample-data presents a “left-skewed distribution”, and the data on the left side of the mean is less than the data on the right side; a smaller absolute number value indicates that although the data distribution is uneven, the overall difference is not large. The kurtosis value is −1.2458, indicating that the overall sample data is relatively flat. This means that the level of GIE is very stable, and maintains a steady and progressive development trend.

③. Pertaining to the distribution of resources and the company's time-period., the mean and median are very close, and the absolute-values of “skewness and kurtosis data” are very small. This implies that the overall data presents a more “symmetrical distribution”. At the level of development potential, the skewness value of the sample data is 3.1969, indicating that the overall sample-data presents a “right-skewed distribution”. The data on the right side of the mean is less than the data on the left side, and there are a few sample companies whose Tobin-Q values are larger, with the maximum value reaching 10.1589. The mean and median of the data are relatively close, and the “standard deviation of the data” is small, indicating that the difference between the data is small.

RETRACTED

#### 4.3.2 Cointegration test based on panel data

After concluding that second-order single integration exists in panel data, further test whether the co-integration relationship exists in panel data. Kao (1999) test was used to conduct “co-integration test”, and the test outcomes at the significance level of 1% rejected the original-hypothesis that there is no “co-integration relationship”, so it can be considered that there is a co-integration relationship in panel data [21].

It is indeed the p-values in parentheses in Table 3 that are indicated. A statistical measure that assesses the strength of proof opposing the null hypothesis is the p-value. To be more precise, it establishes whether the variables under analysis have a cointegration relationship. If the p-value is lower than the significance level, it provides strong demonstrate opposing the null hypothesis (in this case 0.01), which suggests that the alternative hypothesis (that a cointegration relationship exists) should be considered.

**Table 3:** Cointegration test results for correlated variables.

Testing method	RE investment and GIE level	RE investment and GIE level and other control variables
“Panel PP”	“-8.0826” “(0.0000)”	“-3.1275” “(0.0009)”
“Panel ADF”	“-11.7690” “(0.0000)”	“-2.9774” “(0.0015)”
“Group PP”	“-8.8801” “(0.0000)”	“-10.2553” “(0.0000)”
“Group ADF”	“-12.3452” “(0.0000)”	“-5.2328” “(0.0000)”

As a result, the p-values in Table 3 indicate that the variables being tested exhibit a cointegration relationship. In particular, all p-values are less than 0.01, strongly supporting the null hypothesis for all tests and combinations of variables. Table 3 is the test results of related variables.

The outcomes in Table 3 show that there is a relatively stable relationship among the factors.

#### 4.3.3 Test of nonlinear effect

##### 4.3.3.1 Construction of the model

Considering that the semi-parametric method is a method between the parametric model and the non-parametric model, it has the following advantages: Firstly, it can not only eliminate the problem of improper model setting that may exist in the parametric model, but also prevent the “dimensional bane” problem that the non-parametric model may bring. Therefore, the semi-parametric model has high estimation efficiency for parameters and good interpretability for data modeling [22,23]. Secondly, in general, scholars solve nonlinear problems by linearizing nonlinear problems and then using linear models to deal with them. However, some nonlinear problems cannot be obtained satisfactory results through linearization because the model is set to the nonlinear form [24]. The semi-parametric estimation theory can effectively solve the model setting problem with strong nonlinearity [[25], [26], [27]].

RETRACTED

##### 4.3.3.2 Analysis of empirical test results

The model was modified by stepwise regression. Table 4 shows the outcomes of the GIE for investment in RE.

**Table 4:** Benchmark model estimation results for GIE and RE investment.

test variable	estimated value	standard error	T-statistic	P-value
“RE”	“1.08″	“0.32″	“3.35″	“0.00″
“AGE”	“-0.02″	“0.12″	“-0.20″	“0.84″
“TQ”	“-0.71″	“0.07″	“-10.91″	“0.00″
“G (INDEX)”	“/”	“0.42″	“-1.74″	“0.08″

Among them, the solid line in Fig. 7 exhibits the “non-linear relationship”, and the dotted line is the confidence interval.

**Fig. 7:** Nonlinear relationship.

It can be seen from Fig. 7 that it is found that the “W”-type nonlinear relationship actually means that the relationship between the two is unstable, sometimes positive and sometimes negative. The reason is that the policies contained in the GIE system are very complicated [[28], [29], [30]]. In addition to the government's green subsidies, green credit, and environmental tax policies as the main channels, there are also an immense policies that have not been executed [[31], [32], [33]]. On the one hand, these policies develop slowly and are strongly influenced by the government's will, so they are extremely unstable; on the other hand, when they play a role, they can present a state of mutual game, which may amplify, weaken or even offset the effects of policies.

From the perspective of the role of control variables, since the enterprise resource endowment is selected as an inverse index, the enterprise resource endowment may significantly inhibit the level of RE investment. Most of the highly-developed venture companies can use creditor funds to apply high-efficient production and operation. In addition to blind borrowing behavior, the debt ratio of enterprises has been imperceptibly and has an indicative significance to show the vitality of the enterprise [[34], [35], [36]]. Most of the venture companies with high debt-ratio, that is, insufficient resource endowment, have a strong sense of competition and more aggressive business strategies. This shows that RE companies should adequately rise the debt-ratio in exchange for higher profit-space, and enhance the business-vitality of the company.

RETRACTED

Fig. 8 shows the grouping estimation results of the constituent elements of different layers.

**Fig. 8:** Relationship between different factors and investment in RE.

In the GIE system, the supervision and disclosure system are shown in Fig. 8(a); the normative system is shown in Fig. 8(b), and the green accounting system is shown in Fig. 8(c). Although the development of the green supervision and disclosure system and the green accounting system has yet to be perfected, specifically, most policies still have problems such as “alternative implementation”, “perfunctory implementation” and “contradictory implementation” in the process of implementation, so that the implementation of policies has not yet been implemented, and a series of policies promulgated under the green supervision and disclosure system mainly supervise the green behavior of enterprises at the pre-control level, which can effectively reduce or even avoid the occurrence of environmental pollution behaviors from the “source”. Therefore, the government generally attaches great importance to the implementation of policies at this level and implements them more vigorously, so it has a strong role in promoting investment in RE. Incorporating environmental data into the accounting system from a post-accounting perspective is the goal of the green accounting system. This offers the nation accurate green economic information [37,38]. Although the policy development prospects at this level are promising, it has just entered the public eye in recent years and needs to go through a long process. At the same time, the government's attention needs to be strengthened, and the impact on RE investment has not yet appeared.

A complex non-linear relationship between the green regulatory system and the investment in RE has an impact. The reason for this is that, firstly, although the policies promulgated at the level of prior control are very important, since the government is aware of the negative consequences of ongoing pollution and irreversible resource depletion, it places a high priority on environmental governance practices during production. Secondly, due to the high importance of the state, and a large number of policies under the green standard system were introduced earlier and the implementation process was long, the development of the green standard system could be more perfect.

RETRACTED

### 4.4 Examination of the role of GIE in influencing RE Investment—the perspective of industry and enterprise heterogeneity

Considering the heterogeneity of industries and enterprises, this section intends to explore the effect of industry heterogeneity and enterprise size differences on the nonlinear relationship between GIE and RE investment. The research conclusions are of great significance for promoting the coordination and cooperation among various policies in the system and the effect game, coordinating the development of RE enterprises among industries, and objectively locating the focus and direction of policies.

#### 4.4.1 Based on the perspective of industry heterogeneity

Based on this, the model is estimated, and the results show that there is a linear relationship between the level of GIE and RE investment in different industries, as shown in Fig. 9.

**Fig. 9:** The relationship between the level of GIE and RE investment in different industries.

As can be seen from Fig. 9, the impact of the GIE level on RE investment presents obvious industry differences. Fig. 9(a) is the impact of the GIE on the solar energy industry, and Fig. 9(b) is the impact of the GIE on the hydropower industry. Specifically:

①. At the 10% significance level, the GIE level has a promotion coefficient of 1.0697 on the investment in the solar-energy industries. This shows that the GIE can greatly facilitate/encourage the progressive growth of the solar industries.

②. The impact of the GIE level on the investment in the hydropower industry has not passed the significance test. This is mainly because, firstly, the government pays less attention to the industry and the implementation of policies is weak; secondly, its own development conditions are limited. As far as the hydropower industries are concerned, although the hydropower industry has developed early and is rich in resources, its development has been stagnant due to the long-term influence of natural factors that can have an implication on various aspects include “geographic location”, and “climate change”.

#### 4.4.2 Based on the perspective of enterprise-scale differences

Considering the considerable disparities in the development scale of diverse RE enterprises, the 92 RE sample enterprises are divided into “76-large enterprises”, and “16-small and medium-sized enterprises”, and the models are estimated respectively. The results show that there is a linear relationship between the level of GIE and RE investment of different enterprise scales, as shown in Fig. 10.

**Fig. 10:** The relationship between the environmental level of green institutions and RE investment by different types of enterprises

Fig. 10(a) is the relationship between the level of GIE and RE investment of large enterprises, and Fig. 10(b) is the relationship between the level of GIE and RE investment of small, medium, and micro enterprises. It can be concluded that at the 1% significance level, the GIE level has a promotion coefficient of 1.8276 on the RE investment of “small and medium-sized enterprises”. The impact on large-scale corporate RE investment failed the significance test. A company's ability to raise capital and develop its business strategy is influenced by its size. Large businesses benefit from economies of scale and scope, which increases their management, risk-taking, and financial flexibility. They are less dependent on government regulations and have a variety of funding options. Small and medium-sized micro-enterprises, on the other hand, struggle with funding and have a lack of resources, leaving them largely dependent on government regulations and their sensitivity is higher [39,40]. Therefore, the promotion effect of the GIE level on its investment behavior is more obvious.

RETRACTED

### 4.5 Discussion and countermeasures

#### 4.5.1 Discussion of experimental results

The empirical test results indicate that there is a non-linear relationship between investments in renewable energy and green institutional environments. This relationship is shaped like the letter “W,” showing a two-way impact of the green institutional environment on renewable energy. Depending on the strength of these two effects, the direction in which the green institutional environment level affects investments in renewable energy is determined.

#### 4.5.2 Countermeasures and suggestions

The green institutional environment plays an important role in supporting the development of renewable energy. Therefore, to maintain the positive impact of the GIE on RE investment, the government should, on the one hand, give full play to its policy-leading role, and actively guide and stimulate greater awareness of social capital and renewable energy companies. On the other hand, to encourage investment, it is necessary to give full play to the core role of the green institutional environment, ensure its rationality, avoid over-implementation of policies, and maintain the stability and continuity of macroeconomic policies to create a healthy and sound environment. Green institutional environment and avoid drastic fluctuations in the policy environment affecting the development of the renewable energy sector. For enterprises, renewable energy enterprises should maintain a good corporate image, eliminate social capital financing obstacles, and reduce financing costs. Enterprises should also focus on improving their own capital supervision mechanisms, ensuring the use of capital channels, and maximizing the efficiency of capital use.

RETRACTED

#### 4.5.3 Deficiencies

This paper examines in detail the implications of a GIR on RE investment and presents findings that complement previous research. However, there are still several issues to be discussed: First, many policies and systems have not been implemented before and after the fact, and the information disclosure mechanism is unreliable. Some indicators are also difficult to obtain or inconsistent; second, this paper integrates different environmental and economic policies policy, and explores the non-linear direct impact of the GIE on RE investment.

## 5 Conclusions

In today's world, whether it is industry, agricultural production, or the normal living needs of ordinary people, energy consumption is inseparable. The ability to effectively develop energy, utilize energy efficiently, and the per capita availability of energy are currently important indicators to measure a country's production and creativity capabilities and people's living standards. Through the investigation and research on RE and energy efficiency financing, the results showed that the level of GIE played had a significant role in promoting investment in the solar energy industry. This showed that the government attached great importance to the development of the solar energy industry, and the GIE created could greatly promote the development of the solar energy industry. For the hydropower industry, the impact of the GIE on the investment in the hydropower industry was not significant, indicating that, on the one hand, the government's attention needed to be strengthened. On the other hand, the government should provide targeted help according to the development characteristics of each industry as much as possible. The level of GIE had a significant role in promoting RE investment in small and medium-sized enterprises, while the impact on RE investment in large enterprises did not pass had not passed the significance test. This showed that the GIE had strong support for small, medium and micro enterprises, but not much help to large enterprises. For To the lack of specific practice of the research theory, there is still a long way to go.

With the development level of modern science and technology and the continuous improvement of human life quality requirements, the energy demand demand for energy is increasing sharply, accelerating the consumption rate of fossil energy such as oil, natural gas and coal, making the total surplus of fossil energy in the world constantly reduced, and the future social and economic development is faced with a direct energy shortage problem. We need to adhere to the path of green and low-carbon development that gives priority to ecology, accelerates the adjustment of the energy mix, and promotes green and low-carbon reform of energy production and consumption patterns. Future research directions should focus on the following issues: First, the green institutional environment involves many different fields. The second is to optimize the selection of environmental evaluation indicators for the green system, and to find efficient and easy-to-obtain data. Third, based on the basis of the existing research results, the impact of political games on the green institutional environment and the indirect impact on enterprises' investment in renewable energy should be further investigated through appropriate channels. This paper hopes to keep up with the situation in the future and make further development by combining green regeneration and artificial intelligence.

RETRACTED

## Author's contributions

Author (1) Conceived and designed the experiments; Performed the experiments; Wrote the paper. Author (2) Conceived and designed the experiments; Performed the experiments; Wrote the paper. Author (3) Conceived and designed the experiments; Performed the experiments; Wrote the paper. Author (4) Conceived and designed the experiments; Performed the experiments; Wrote the paper. Author (5) Analyzed and interpreted the data; Wrote the paper; Critically revisions of the paper. Author (6) Conceived and designed the experiments; Performed the experiments; Analyzed and interpreted the data; Wrote the paper. Author (7) Performed the experiments; Analyzed and interpreted the data; Wrote the paper; Critically revisions of the paper. Author (8) Performed the experiments; Analyzed and interpreted the data; Wrote the paper. Author (9) Performed the experiments; Analyzed and interpreted the data; Wrote the paper.

## Funding

This work has received no external fundings.

## Data availability statement

Data included in article/supp. material/referenced in article.

## Declaration of competing interest

The authors declare that they have no known competing financial interests or personal relationships that could have appeared to influence the work reported in this paper.

## Appendix A Supplementary data

Authorship-Change-form renewable energy Authorship-Change-form renewable energy
